# How Do Green Finance and Energy Efficiency Mitigate Carbon Emissions Without Reducing Economic Growth in G7 Countries?

This article has been retracted.

**DOI:** 10.3389/fpsyg.2022.879741

**Published:** 2022-05-03

**Authors:** Zhen Fang, Can Yang, Xiaowei Song

**Affiliations:** ^1^School of Management, Ocean University of China, Qingdao, China; ^2^SINOTRUK Finance Co., Ltd., Jinan, China

**Keywords:** energy conversion, energy efficiency, green finance, environment protection, financing efficiency

## Abstract

Climate change is one of the most serious threats facing the world today. Environmental pollution and depletion of natural resources have been highlighted by the United Nations Sustainable Development Goals (SDGs), paving the way for modern concepts such as sustainable growth to be introduced. Therefore, this research explores the relationship between green finance, energy efficiency, and CO_2_ emissions in the G7 countries. The study uses panel data model technique to examine the dependence structure of green finance, energy efficiency, and CO_2_ emissions. Moreover, we use DEA to construct an energy efficiency index of G7 countries. A specific interval exists between the values of the energy efficiency indexes. Japan, the United Kingdom, and the United States were named the most energy-efficient countries in the world, based on results obtained for five consecutive years in this category. However, according to the comparative rankings, France and Italy are the most successful of all the G7 members, followed by the United Kingdom and Germany. Our overall findings of the econometric model confirm the negative impact of green finance and energy efficiency on CO_2_ emissions; however, this relationship varies across the different quantiles of the two variables. The findings in the study confirm that green finance is the best financial strategy for reducing CO_2_ emissions.

## Introduction

The burning of fossil fuels, according to environmental scientists, is the primary reason for greenhouse effect (Ahmad et al., 2021; Abbasi et al., 2022). Greenhouse effect is the buildup of heat in the atmosphere (Ali et al., 2021; Hao Y. et al., 2021; Iqbal et al., 2021b). An important consideration in making any decision is a country’s economic growth is the amount of energy it uses (Islam et al., 2021; Ahmad et al., 2022; Irfan and Ahmad, 2022; Irfan et al., 2022). Excessive use of energy, on the other hand, leads to atmospheric emissions of CO_2_, SO_2_, and CH_4_ that degrade the environment (Khan I. et al., 2021; Rauf et al., 2021; Nuvvula et al., 2022). To strike a balance between environmental damage and energy security, restrictions imposed by both the economy and the environment have a role (Tanveer et al., 2021; Wu et al., 2021; Wen et al., 2022). Rapidly rising power demand and prices, resource scarcity, and the social and political consequences of global warming have all contributed to a significant increase in energy security (Razzaq et al., 2020, 2021; Shi et al., 2022). Similarly, rapid economic growth is one of many factors driving up global energy consumption, which has in turn created significant environmental concerns around the world (Yang et al., 2020; Irfan et al., 2021b,c; Xiang et al., 2022). To put it another way, G7 countries account for a disproportionate amount of global warming and climate change. A small number of countries have made only the bare minimum effort to reduce global average temperatures, despite their small size (Tang et al., 2022). Many countries lack the financial resources to generate electricity from renewable sources of energy because of their massive economies’ ever-increasing demand for energy (Irfan and Ahmad, 2021; Irfan et al., 2021a). Because of this, rising temperatures are impacting the environment in a bad way.

With the glaciers disappearing and the level of sea rising due to climate change, the hands of time seem to be counting down (Irfan et al., 2020; Elavarasan et al., 2022a,b). More and more people are dying as a result of floods, droughts, heat strokes, and other natural disasters (Elavarasan et al., 2021; Yan et al., 2021). Arctic A threefold increase in heat has been observed in Canada, while temperatures have risen by more than two degrees Celsius over the global average (Li et al., 2021; Hou et al., 2022). People’s homes are being destroyed, food is becoming scarcer, and ravenous animals such as bears are on the loose because of the melting of the glaciers. A total of 200 people lost their lives in Japan in 2018 due to landslides and floods caused by the country’s record-breaking rainfall. Unimaginable heat waves also threatened the region’s most vulnerable species. Extreme weather events will become more frequent and more severe as a result of climate change, and the region’s energy consumption will more than double from its current level (Jin et al., 2021; Wang and Luo, 2022). Japanese continuing construction of coal-fired power stations is regrettable. Japan’s megabanks have spent $186 billion on fossil fuels since the Paris Agreement was signed, showing that the country’s approach to climate change and global warming is worrying. It is possible that 143 million people who have been affected by the effects of climate change will seek refuge in developed countries.

G7 recent progress in creating green financial markets and a green financial system has raised some questions about the role of green finance development in promoting green productivity. Green finance has emerged as a key tool in the green economy transformation. This year’s total green bond issuance was US$55.8 billion, accounting for 22% of world issues, according to the Climate Bond Initiative (CBI) (Abbas et al., 2020, 2021; Iqbal et al., 2021c; Zeng et al., 2022). Interest in green finance and its impact on economic and environmental sustainability has grown in recent years, as green finance has become more widely available (Zhou et al., 2020; Dmuchowski et al., 2021; Saeed Meo and Karim, 2021; Wang et al., 2022). The impact of green finance development on green productivity research cannot be understated, as it is a major source of green bonds issuance around the world. Using green finance’s capital support function to expedite adjustment of the economic structure and enhance the quality of supply-side investments can help stabilize the growth of the economy from a purely economic standpoint. Sustainable economic and environmental development can be achieved by utilizing the “going green” feature to direct businesses green innovation, environmental protection, and corporate social responsibility and environmental performance (Ahukaemere et al., 2020; Yu et al., 2022).

The current study’s contributions are summarized as follows: In the first place, we fill a void in academic report by examining the link between green finance, energy efficiency, and environmental degradation. The development of green finance is a significant influencer. Energy efficiency in contrast to the green productivity is typically measured in terms of scale, technology, and structure; this is a common approach to measuring green productivity. As a result, a better understanding of the factors influencing green productivity can be gleaned from the financial as well as the real estate industries. For a clearer picture of the job of green finance in the green economy, we introduce comprehensive low-carbon financial flows and investment in environmentally friendly products and services are just two of the many ways to measure the impact on climate change from a more holistic perspective. In terms of green finance, the use of a multidimensional index could result in a more comprehensive evaluation of its development. Third, we use them to address the potential omission of energy and environmental constraints, a super-SBM model with undesirable output has been developed, in contrast to previous productivity studies that primarily focused on good output.

The rest of the document is organized as follows: To begin, section “Introduction” provides an overview; section “Literature Review” details the data and methodology; section “Methodology and Data” provides an overview of the findings; and section “Results and Discussion” concludes the study.

## Literature Review

### The Concept of Green Finance

Finance for, on the other hand, climate change adaptation and mitigation are important provided. However, green finance encompasses not only climate finance, but also a wider range of financial services and products that are focused on a wide objective for the environment such as pollution control, conservation of biodiversity, and natural recourses preservation. However, since its inception in 2010, the Green Climate Fund (GCF) has provided financial assistance to developing nations so that they can better prepare for and cope with the effects of climate change (Pan and Chen, 2021; Zhang et al., 2021a). It was also identified that green finance is essential to financing climate change action following the adoption in 2015 of the Paris Agreement and the Sustainable Development Goals (SDGs) and Sendai Framework for Disaster Risk Reduction (DRRR) (Truby et al., 2022). Various public and private financial institutions are a part of this, along with a variety of asset classes such as “green bonds,” “green loans,” “green funds,” “green banks,” and “green credits,” as well as “climate finance,” “environmentalism,” “carbon finance,” “sustainable finance,” and “sustainable bonds (Wang and Dong, 2022).” Green financing is clearly as a climate change mitigation strategy for green buildings strategy in the building sector. GF-in-GBs will be discussed in depth in the sections that follow, as well as suggestions for how it can be applied better in the future in terms of research, policy, and clinical practice (Huang et al., 2021; Latif et al., 2021; Liu et al., 2021; Mohsin et al., 2021).

### Green Finance and Environmental Performance

Effects of financial assistance, resource allocation, and technological advancement, and so on are just a few of the ways that green finance can influence environmental performance. The capital support effect shows that it is possible to achieve better environmental performance by using Low-energy, low-pollution, and low-carbon emissions are the goals of green finance while also discouraging high-pollution and high-emission production behavior. According to Srivastava et al. (2021), the creation of a green credit policy in the People’s Republic of China affects the financing costs of enterprises. For high-emission and high-pollution businesses, green credit raises the cost of financing, while it lowers the cost of financing for environmentally friendly businesses, according to their empirical findings. van Veelen (2021) examines the macro-mechanistic role of development of green finance and the effects of green finance on the eco-system is examined. According to the researchers, the impact of green finance varies by region on ecological efficiency.

For example, green finance has the ability to increase capital efficiency and redirect the redirection of financial resources from inefficient and polluting operations industries toward more efficient ones, thereby promoting industrial upgrading, optimizing the energy structure of the economy, and improving the quality of life in the surrounding area. On the basis of micro-mechanics discovered, Zhang et al. (2021b) investigate the impact of a green-credit policy on the loan performance of enterprises. Findings suggest that refusal businesses are credible to pay higher interest rates and have a more difficult time securing loan because of this. In order to improve environmental quality at the macroeconomic level, a well-developed financial system can help alleviate financial constraints on environmentally friendly businesses and promote green upgrading.

This innovation effect in technology means that green finance can help companies that are pursuing green technology innovation obtain external credit, thereby reducing energy consumption while simultaneously promoting growth in the green industry and reducing environmental damage and pollution. Toward this end, Khan M. A. et al. (2021) developed a green loan theory that incorporates the interests of businesses, banks, and the government. It is concluded that government subsidies can lower the cost of financing for businesses, increasing the likelihood that they will implement technological innovation. For high-polluting enterprises, Iqbal et al. (2021a) investigate the influence of a green credit policy on green innovation. A statistically significant increase in green patents was found to be a result of the implementation of the “Green Credit Guidelines” in 2012.

## Methodology and Data

### Energy Efficiency

Both the energy economics and environmental index have The DEA non-parametric frontier approach has been used to build the model, which was first introduced by Lozano and Gutiérrez (2008) and later developed further by Mostafa (2011). Slack-based models are being used broadly in a wide range of energy and environmental studies today. Frequently, corporations prioritize beneficial output maximization over model efficiency maximization, while they are equally concerned with minimizing nasty output minimization. At the same time, the manufacturing process is unavoidably enriched by a wide range of contaminants and wastes, including greenhouse gases and other forms of contamination. Maintaining a healthy balance between environmental performance and growth in the economy are linked is essential. Let n be the number of components of the energy vector, economic and environmental variable with entity. A common practice in developing the EVI to rank environmental performance of numerous entities, each underlying entity is ranked according to an environmental index, which can be differentiated from one another by the choice of ordering based on Rn. EVI can also be developed using the mapping function I = Rn→R, which may meet the following condition:


(1) $${\text{V}}_{\text{k}}≽{\text{V}}_{\text{l}}\Leftrightarrow I\,\left({\text{V}}_{\text{k}}\right)\geq I\,\left({\text{V}}_{\text{l}}\right)\,\forall k,l\in \left\{1,\ldots ,K\right\}$$

Conversion functions are used to show how the basic units n-factored evaluation can be changed as:


(2) $$F:\left(V_{\mathrm{k1}},\ldots ,{\text{V}}_{\text{kn}}\right)\to \left({\text{f}}_{1}\,\left({\text{V}}_{\mathrm{k1}}\right),\ldots ,{\text{f}}_{\text{n}}\,\left({\text{V}}_{\text{kn}}\right)\right)$$

When it comes to the extension, the acceptable transformation is involved in this manner as stated by Galvão et al. (2011) and Son et al. (2014) that satisfies, according to EVI, a series of numerous fundamental entities, each of which is expected to elect invariant, is used to evaluate the acceptable transformation of the underlying indicators in order to construct an EVI index for economic, energy, and environmental indicators in each of the three categories.


(3) $${\text{V}}_{\text{k}}≽{\text{V}}_{\text{l}}\Leftrightarrow F\,\left({\text{V}}_{\text{k}}\right)\geq F\,\left({\text{V}}_{\text{l}}\right)\,\forall k,l\in \left\{1,\ldots ,K\right\}$$

Using a ratio scale and only positive variables, this study (Rasoulinezhad and Taghizadeh-Hesary, 2022) found that the geometric mean produced an important index, proving the geometric mean’s significance. In order to quantify alternative aggregation procedures for the development of energy and environmental indices, Ye et al. (2022) developed criteria for estimating information loss. It was also described in detail how Liu et al. (2021) developed the non-compensatory aggregation method, including its use in energy and environmental studies. In addition to the normalization and aggregation of data, a variety of other studies are conducted using composite indicators and weighting.

The DMU0, on the other hand, is efficient if pollution-free environmental efficiency is the primary goal of the study. When it comes to creating an environmentally friendly DMU0, model number 4 is used, primarily for assessing economic efficiency using the SBM model, which utilizes DMUs’ common input and output variables. DMU0 is only efficient when slacks are equal to zero, and only in this case does model 3 meet this requirement. It generates environmental efficiency values when model no 2 is used, while model no 3 generates economic efficiency values when an optimal adverse output from model no 2 is used as a fixative level. According to the findings of Chen et al. (2021), the combined index developed by the researchers can be used for both environmental and economic efficiency modeling. Even though these efficiency values were replicated, the process of obtaining this score has been lengthy. A non-parametric approach in conjunction with linear programming was used in this study to create an index of energy efficiency (EEE) by calculating the average sum of the binary efficiency values. With this, we can classify the most effective frontier practices and assess the relative performance of each of the underlying indicators in light of inputs and outputs from comparable and quantifiable sources (Nawaz et al., 2021).

To demonstrate the systematic productivity and performance of various objects or decision-making units, researchers have turned to data envelopment analysis (DEA), also known as DEA assessment (Bhuiyan et al., 2018; Zhang et al., 2022). It is used to evaluate energy and environmental performance by taking into account the difference between desirable and undesirable outcomes. Zhou et al. (2022), laid the groundwork for the acceptance of a non-parametric DEA frontier practice to measure the undesirable outputs of energy and environmental performance. To distinguish between certain output and input variables, the underlying vectors of variable are exchanged through another set of underlying variables X k,Y k = (xk1,⋯,xkm,yk1,⋯,yks) are both input and output vectors. This has the effect of reducing the amount of primary energy used. 20% of the energy consumption can be saved if the DMU’s value equals 80% (Xiong and Sun, 2022). An assessment of energy and environmental techniques (Guo et al., 2022) is the sole focus of this article. For example, the efficiency of energy-related emissions is measured by Li et al. (2022). To improve environmental performance, Saeed Meo and Karim (2021) offer an SBM measure that uses poor output as an input. As long as you have input vectors that can be used to produce a certain level of output vectors. There is a plethora of possible input-output combinations when X∈ and outputs X∈ are used together.


(4) $$\text{S}=\{\left(X,Y\right):S=\sum_{k=1}^{K}x_{\text{ik}}{\text{z}}_{\text{k}}\leq x_{i,}\;i=1,\ldots ,m$$

$$\text{S}=\sum_{k=1}^{K}{\text{y}}_{\text{rk}}\,{\text{z}}_{\text{k}}\leq x_{r,}\;\text{r}=1,\ldots ,S$$

$$\text{S}=\sum_{k=1}^{K}{\text{z}}_{\text{k}}=1,\text{i}=1,\ldots ,m$$

$${\text{z}}_{\text{k}}>0,k=1,\ldots ,K\}$$

In contrast to Model 4, which only modifies CO_2_ emissions, Model No. 5 modifies all negative outputs. This can be seen by comparing Model 4 to Model 3. Furthermore, the author emphasizes the importance of Model No. 4, which is the DEA model with an adverse output placement (Zhang et al., 2021b). The method considers the inability to effectively deal with the undesirable output when processing the desired and undesirable outputs in that order. On the contrary, it treats each and every one of its inputs as if they were all identical.

max $\frac{1}{m\,s}\,\left(\sum_{k=1}^{K}\frac{{\text{S}}_{\text{i}}^{-}}{{\text{R}}_{\text{i}}^{-}}\,\sum_{k=1}^{K}\frac{{\text{S}}_{\text{r}}}{{\text{R}}_{\text{r}}}\right)$


(5) $$\text{S}=\sum_{k=1}^{K}x_{\text{ik}}\,{\text{z}}_{\text{k}}\,{\text{S}}_{\text{i}}^{-}=x_{0\,i},i=1,\ldots ,m$$

$$\text{S}=\sum_{k=1}^{K}{\text{y}}_{\text{rk}}\,{\text{z}}_{\text{k}}-{\text{S}}_{\text{r}}^{-}={\text{y}}_{0\,r},r=1,\ldots ,S$$

$$\text{S}=\sum_{k=1}^{K}{\text{z}}_{\text{k}}=1,i=1,\ldots ,m$$

$${\text{z}}_{\text{k}}>0,{\text{S}}_{\text{i}}^{-}>0,{\text{S}}_{\text{r}}^{-}>0$$

### Econometric Estimation

The estimations are made using a panel country fixed-effects model. Countries’ fixed effects (i.e., unobservable factors) are shown in Eq. (1). All the time-invariant variations between countries are accounted for by the country fixed effects (such as cultural factors). To be clear, panel fixed-effect models are frequently employed in studies examining the causes of air pollution. The first model is written as:


(6) C⁢O2i⁢t=β1⁢G⁢Fi⁢t+β2⁢E⁢Ei⁢t+β3⁢Xi⁢t+vi⁢t+ui⁢t

where is CO_2_ emissions of country *i* at year *t*; *GF* represents green finance index and includes the current as well as one lag of this index; is the energy efficiency of country *i* at year *t and X* is a vector of control variables; *v*_*i*_ is the country-fixed effects; *i* = 1, …, n denotes the country; and *u* is the error term.

All variables, with the exception of the energy efficiency index, renewable energy consumption, and urbanization rate, are transformed into logarithmic values for the purposes of estimation and forecasting. Detailed descriptive statistics (mean and standard deviation) for the variables are provided in Table 1.

**TABLE 1:** Descriptive statistics.

Variable	Mean	Std. Dev.	Min.	Max.
EE	0.52	0.698	0.446	1
GF	0.302	0.0746	0.159	0.621
PGDP	10.13	0.576	8.528	11.53
RE	94.98	40.65	3.8	242.3
URB	54.11	13.65	27	90
IND	38.74	8.484	11.84	53.04
TRADE	30.34	36.54	1.69	172.2
FDI	2.258	1.728	0.01	8.19
EDU	8.829	0.985	6.59	12.68
R&D	1.47	1.061	0.2	6.01

## Results and Discussion

### Energy Efficiency

Although the specific trend of German CO_2_ emissions has become significantly higher than the common trend over the past few decades, it follows the common trend. Finally, average trends are increasing and emissions in Italy are trending horizontally. For instance, most developed countries seem to converge at the highest peaks, except for Canada and France, which seem to have a different path to efficiency, even though they started to be the most energy-consuming countries during this period. Fossil energy processes, which produce large amounts of carbon dioxide emissions, were largely responsible for the majority of global economic growth in the twentieth century. According to policymakers, any reduction in carbon dioxide emissions will have an adverse effect on the economy. The economies of major countries continue to struggle even with reduced emissions. like the United States can grow their GDP and their economic output, but pollution does not have to rise at the same time. This is based on new subjective evidence, however. That’s because industries and economies are moving away from large energy-intensive technologies and toward smaller ones. Between 0.65 and 0.70 is a structural shift, efficiency, and the typical intensity of energy index Structural reallocation has resulted in an increase in energy intensity and a decrease in their energy efficiency. Table 1 contains the individual indicator score of G7 economies. Shocking eco-friendly concerns, like a global warming, are connected with the use of abundant energy utilization because of prompt growth and development (Yao and Tang, 2021). This study employs the DEA models to assess the efficiency of energy consumption, environment-economy and CO_2_ emissions for the G7 economies, the efficiency of energy use and CO_2_ emission efficiency, separately, and economic efficiency and environmental efficiency. These pursue an equilibrium between the economic development and environmental performance of a country However, the comparative rankings indicate that France and Italy are the best amongst all considered members.

Energy concentration cannot be used to assess the efficiency of any country’s energy consumption, as can be seen from a comparison of the two concepts’ relative effectiveness in terms of energy consumption and concentration. Consequently, France and Italy were recognized as equally competent and well-performing countries during the periods, whereas Japan, Canada, and the United States are the last three economies among all G7 members for almost every year with respect to CO_2_ emission efficiency. For all G7 countries, the efficiency scores are less than 0.50 for emission efficiency of CO_2_, enlightening greatly significant variances among G7 economies in emission efficiency of CO_2_. Additionally, the majority of G7 countries’ research studies have greater points in environmental economic efficiency as compared to CO_2_ emission efficiency, where Canada and France are the only two exclusions. Japan and France are the two milestones and bench-marking markets that were recognized as efficient in both CO_2_ emissions and energy consumption. Considering a greater extent of economic and environmental efficiency, it is concluded that the majority of the G7 countries demonstrated better economic efficiency as compared to environmental efficiency. When studying the relationships between energy consumption efficiency and emission efficiency of CO_2_, the study concluded that energy consumption efficiency and emission efficiency of CO_2_ can help to decrease environmental condition.

This was achieved by assessing the environmental and energy equity. The energy intensity and environmental index analysis shows the best score, where the United Kingdom and the United States are the two countries with the worst results. For countries, maintaining economic development without affecting energy utilization is quite challenging -the development of energy-related efficiency in the world’s major economies, while reducing energy waste and pollution Taghizadeh-Hesary et al. (2021) concluded that energy consumption and economic growth are directly related to energy and environmental efficiency.

Table 2 shows energy intensity and energy efficiency scores. In this study, energy, economy, and environmental indicators are used to measure energy, economic, and environmental efficiency and CO_2_ emissions. The G7 countries’ economic and environmental efficiency scores show the best undesirable output should be fixed to generate an economic efficiency score for environmental efficiency. In general countries with greater economic and environmental efficiency, according to the findings scores have a more efficient economy and environment than countries with lower economic or environmental efficiency scores. There are two countries in the world that are less efficient than France and Canada.

**TABLE 2:** Energy efficiency of G7 countries.

	2010	2011	2012	2013	2014	2015	2016	2017	2018	2019
Canada	0.51	0.45	0.49	0.41	0.55	0.59	0.55	0.68	0.49	0.63
France	0.88	0.87	0.94	0.88	0.97	0.93	0.88	1	1	1
Germany	0.47	0.45	0.41	0.51	0.37	0.44	0.26	0.34	0.33	0.38
Italy	0.88	0.82	0.86	0.77	0.69	0.77	0.72	0.66	0.74	0.76
Japan	0.52	0.54	0.61	0.45	0.26	0.26	0.21	0.24	0.19	0.22
United Kingdom	1	1	1	0.99	1	1	0.98	1	0.95	0.98
United States	0.46	0.45	0.41	0.46	0.34	0.35	0.37	0.39	0.37	0.39

### Econometric Estimation

The fixed effects are shown in Table 3. It appears that green finance development can increase the level of green productivity at the 5% level, based on GF coefficients as the primary explanatory variable. There is strong evidence it is possible to achieve a win-win situation with green investment and credit for both the environment and the economy, which in turn can lead to increased green economic development. As a result, in order to alleviate China’s financial constraints, the country’s central government should focus on this issue alone by businesses while undertaking environmental-friendly activities, which necessitates the development of an operating green financial system. Companies are more likely to do so to get actively involved in green economic development activities if they did this.

**TABLE 3:** Results of fixed-effects regressions.

Variable	OLS	Fixed effect
GF	−0.002	−0.001
	(−0.31)	(−0.029)
EE	−0.019***	−0.133***
	(−7.52)	(−9.31)
RE	0.026**	0.031*
	−1.992	−1.842
GDPpc	−0.007**	−0.111*
	(−2.018)	(−1.327)
Trade	−0.003***	−0.054
	(−4.052)	(−1.342)
Education	0.021***	0.0132
	−3.933	−0.895
R&D	0.012	0.236
	(−0.342)	(−1.358)
Urbanization	−0.007**	−0.009*
	(−2.269)	(−1.843)
Constant	1.022***	1.321***
	−18.55	−19.31
Observations	1,044	698
Firms	98	72
Likelihood	677.22	423.62
Wald chi (2)	543.82	488.42

Significance levels: * = 0.1, ** = 0.05, *** = 0.01.

Evidence shows that most control variables are statistically significant in terms of their influence. The positive correlation between GDP per capita and R&D shows that the more economic progress and technological advancement there is, the greater the potential for increasing green productivity. The findings of Sun et al. (2022) are supported by these findings. However, R&D return the local scientific and technological capabilities that have a positive effect on economic growth Zhang and Vigne (2021). Research and development, on the other hand, can improve the quality of the environment (Huang et al., 2021). The coefficients of trade indicate that the amount of green output decreases with time the structure of how much and how much energy is used in industrialization. We had expected these results, and they confirm our suspicions about China’s excessive urbanization and reliance on coal consumption (Chien et al., 2021; Lee and Lee, 2022; Ning et al., 2022). According to the EDU coefficient, a high degree of traditional education is associated with low green productivity. The wealth effect in emerging economies is to blame for this. To put it another way, a higher level of education tends to lead to an increased demand for energy, which has a negative impact on the environment (Sun et al., 2022).

In addition, 27 percent of coal was used, and there was a noticeable change in 2009 As a result, in 2009, OECD countries reduced their use by around 4.7%, which is on par with the rate in 2000. Sustainable development requires that energy demand be met without compromising the need for environmental protection (Usman et al., 2022). In most cases, the political economy provides a financial foundation for evaluating the degree of energy efficiency in relation to power output per unit. A developing various study are settled in Germany, which have added to activity efficiency of energy by specializing in the analysis of efficiency of total-factor. Whereas, our findings are supported by the study of Hassan et al. (2022). According to these studies, a combination of energy inputs and resources such as greenhouse emissions are used during the combined production process. Zhao S. et al. (2022) evaluated electricity based on a rank-based system. Analysis of energy efficiency in the G7 countries was conducted by Zhang et al. (2022) using Data Envelopment Analysis (DEA) to evaluate the total-factor structure. Economical models require the factors that lead to higher energy performance measures to be taken into account. When Zhao X. et al. (2022) conducted their research to provide environmental upgrading submissions, they relied solely on the investigation of energy potency and the environmental Kuznets curve.

The empirical evidence of this lies beyond the scope of the present study. Therefore, the proposed research study comprises GHG releases, i.e., emissions only for the purpose to unearth the real image of eco-friendly degradation. Renewable energy reduces the environmental deterioration and climate vulnerability (Zahoor et al., 2022). Furthermore, Canada has its energy security and has massive reserves of crude oil, and has vital and effective policies.

### Sensitivity Analysis With Another Measure for Green Finance

The results of sensitivity analysis are shown in Table 4. Equation 1 is re-estimated by replacing the green finance index substituting other proxies for green financing. The total each country’s Climate Bond issue from 2010 to 2019 is known as Climate Bonds. The Climate Bonds Initiative database serves as the source of this variable’s data. An important relationship between GDP growth and greenhouse gas emissions has been found (it caused increase of GHG releases, i.e., emissions with the perspective of Canada due to growth in GDP). GHG emissions, i.e., emissions were positively impacted by the gross domestic product growth that matches, i.e., GDP. When it comes to per capita emissions of greenhouse gases and energy security, countries that use more energy face similar issues as other countries that use more energy (Hao L. N. et al., 2021; Tawiah et al., 2021). Fossil fuel subsidies have been linked to higher GHG emissions and decreased energy security in both developed and less developed countries, according to numerous studies. Furthermore, a number of in both developed and welfare countries, fossil fuel consumption is increasing than their less developed counterparts (Ngo, 2022). Similar strategies are being discouraged because of the growing trend toward renewable energy. In Australia, a reduction in subsidies is expected to reduce GHG emissions by 12 percent by 2030 (Feng and Wu, 2022). According to GHG data, most of the energy consumed in those countries originates in the form of fossil fuel. GHG emissions are lower in countries that use more renewable energy, such as Iceland, which has 77.03 percent renewable energy and “720” GHG emissions. Emissions per kilowatt hour of energy used (Feng and Wu, 2022).

**TABLE 4:** Sensitivity analysis.

Independent variables	(1)	(2)	(3)	(4)
Climate bonds	−0.2702***	−0.1319*	−0.1284*	−0.1933***
	(0.0558)	(0.0769)	(0.0737)	(0.0600)
GDP	1.3807***	0.9317***	0.8345***	1.2642***
	(0.1133)	(0.1896)	(0.2447)	(0.1110)
Population		0.3668***	0.4566**	
		(0.1231)	(0.1810)	
Urbanization				0.6599
				(0.3956)
RE			−1.5191	−0.5514
			(2.112)	(1.0316)
*R* ^2^	0.7356	0.7720	58.77	45.12
*F*-statistic	83.62***	79.19	0.7780	0.7767
Observations	61	61	61	61

Significance levels: * = 0.1, ** = 0.05, *** = 0.01.

### Discussion

In order to the environment and a clear production process must be maintained at all times process and the use of renewable energy are necessary (Dong et al., 2022). Carbon dioxide levels in the atmosphere are expected to rise as a result of an increase in the amount of energy used by industries, according to the study by Dong et al. (2022). This year, CO_2_ concentrations in the atmosphere reached 400 ppm on an annual basis, which is 40% higher than the level in 2016. Emissions of carbon dioxide (CO_2_) have decreased by nearly half since 1980, according to Debrah et al. (2022) and Khan H. et al. (2022).

The United Nations (UN) eco-friendly program is reflected in the energy policies of European countries. A wide range of options are available thanks to new warning technologies and intelligent monitoring. Different and specific methods are recommended to ensure sustainable, environmentally friendly, and crystal-clear production. It is only possible to maintain a clean production through continuous application of a mutually cautious recyclable strategy, which maintains because of its environmental friendliness. Due to the fact that immaculate creation’s application in a wide range of industries, as it necessitates the consumption of the atmosphere’s natural resources (Hu et al., 2022). For example, Proper waste management would be ensured by an efficient environmental management system through investment in research and development. It’s impossible to know how technological advancements will affect carbon emissions without evidence. Because of a rise in economic growth and greater openness to trade, research and development may have an impact on environmental quality, given the positive impact on the expansion and trade of R&D. Energy and environmental efficiency may be enhanced by new technologies, but increased production may still necessitate greater use of natural resources, resulting in higher emissions of CO_2_. As existing knowledge reserves grow, it becomes more difficult to achieve new developments, resulting in lower levels of R&D over time. Economic expansion, on the other hand, necessitates a greater use of natural resources.

Historically, the G7 countries have been larger energy consumers. Various studies on these countries assess their economic growth, energy efficiency, and resilience by considering poor output, energy input, and non-discrimination. However, the contribution of developed countries toward global energy consumption has declined over time. Generally, over the past three decades, the G7 countries have been considered and characterized like the countries with a large industrial volume of production, international gas releases, i.e., emissions, energy utilization, and trade. The goal of this study is to determine how much energy is being used intensity, energy efficiency, and environmental index of these nations, as they contribute entirely a huge volume of releases, i.e., emissions and that is equal to the total worlds’ emissions. Thus, energy consumption is a major concern because of an increase in foreign-imported energy prices. In the meantime, the extensive use of imported oil increases the CO_2_ emission level, which ultimately causes global warming and climate change, decreases farming yield, and threatens human life. In this situation, a new philosophy is a necessity for energy consumption and sustainable economic growth. The logical reason behind selecting the G7 countries is that it shows the divergent results and contains the alarming figure of energy consumption and CO_2_ emission (Hao et al., 2022; Khan I. et al., 2022). Trends in the United States, Canada, and France are usually much higher than the average trends, although CO_2_ emissions in France have converged into a common trend over the past three decades. Japan and the United Kingdom are clearly below the average trend, although UK carbon dioxide emissions have been closer to the average trend in recent decades.

## Conclusion and Policy Implication

Eco-friendly index estimation and alternative methods when it comes to evaluating the effectiveness of energy use and environmental impact are the consequences of the proposed research. With less GHG emissions and renewable energy releases metrics, the lack of efficient environmental performance suggests an overview of GHG’s releases (toxic emissions). Measuring energy concentration and energy efficiency was a perplexing issue that is being faced around the globe to resolve this, an environmental, i.e., eco-friendly index was developed. Keeping in view to construct an eco-friendly index of all G7 nations, applied both arithmetic mean aggregation and DEA, i.e., Data Envelopment Analysis to develop a mathematical aggregation tool. To support the methodology of this study, the standardized EVI was developed by adopting a non-parametric frontier approach. Therefore, in future, further assessment on decision-makers’ preferred weight and rank information may be incorporated. Results of the proposed research work suggest implementing the below recommendations. The main factor of global warming is the utilization of energy; therefore, it must be reduced. Research and development expenditures increase by 1% for every 1% increase costs, Canada, France, Germany, Italy, Japan, and the United States reduce carbon dioxide emissions by 0.18, 0.27, 0.22, 0.09, 0.31, and 0.32%, respectively. In the United Kingdom, a 1% An increase in R&D spending will result in a 0.62 percent increase in emissions, but after accounting for this discrepancy, the effect will be negative. The turning point for valid environmental situations in all countries, except Japan was between $6933 and $36,255.

### We Proposed the Following Policy Framework

• In the short term, these countries may continue to operate at a relatively high level of inefficiency unless their governments change their management style or alter their policies. 1. To put it another way, short-term policies in these economies will increase energy security and carbon emissions. Even though developing countries are making steady progress, developed economies are reluctant to follow suit until their own performance improves.
• It has also been found that by focusing on the economies of each country in the proposed G7 group and comparing their environmental performance, convergence appears to be greater or stronger than it would have been otherwise.
• It is imperative that developing countries take steps to encourage the growth of renewable energy use. Reducing the use of fossil fuels, for example, is an important step toward reducing energy-related carbon dioxide emissions and fostering a green economy. In addition, the growth of fossil fuels should be regulated to ensure sufficient growth. Developing low-carbon energy requires space. The most appropriate and cost-effective way to reduce the environmental impact of energy production is to improve energy efficiency.
• As a result of extreme weather conditions, disasters, and natural disasters, policymakers must increase their ability to resist energy shortages; this would improve energy equity. Oil import risks could be reduced and outdoor oil dependence reduced if energy prices are fixed and not affected by supply and demand or by the use of renewable energy sources.
• Thus, G7 countries should continue to implement innovation-driven approaches and move toward a more enhanced ability to innovate; this can help improve performance by commercializing research and development from G7 nations. Consequently,
• G7 countries play a supporting role for the region’s ecological environment, but the province is the most polluted G7 region. In order to protect their natural environments, countries in South Asia must enforce strict environmental protection legislation and implement shared avoidance, control, and law measures. This would improve environmental quality to the point where it would be more robust to support and guarantee superior economic growth.
• With regard to those who live in cities ranging from small to large have the potential to improve environmental efficiency, although it is expected that industrial transfer demonstration zones will positively contribute.
• In order to reap the benefits of policy-making connected to the industrial transfer demonstration zone, the zone’s policy welfare should be continually improved.

## Data Availability Statement

Data will be provided on reasonable request from corresponding author.

## Author Contributions

All authors listed have made a substantial, direct, and intellectual contribution to the work, and approved it for publication.

## Conflict of Interest

CY was employed by SINOTRUK Finance Co., Ltd. The remaining authors declare that the research was conducted in the absence of any commercial or financial relationships that could be construed as a potential conflict of interest.

## Publisher’s Note

All claims expressed in this article are solely those of the authors and do not necessarily represent those of their affiliated organizations, or those of the publisher, the editors and the reviewers. Any product that may be evaluated in this article, or claim that may be made by its manufacturer, is not guaranteed or endorsed by the publisher.

## References

[B1] AbbasQ.HanifI.Taghizadeh-HesaryF.IqbalW.IqbalN. (2021). “Improving the energy and environmental efficiency for energy poverty reduction,” in *Poverty Reduction for Inclusive Sustainable Growth in Developing Asia. Economics, Law, and Institutions in Asia Pacific*, eds Taghizadeh-HesaryF.PanthamitN.YoshinoN. (Singapore: Springer). 10.1007/978-981-16-1107-0_11

[B2] AbbasQ.NurunnabiM.AlfakhriY.KhanW.HussainA.IqbalW. (2020). The role of fixed capital formation, renewable and non-renewable energy in economic growth and carbon emission: a case study of Belt and Road Initiative project. *Environ. Sci. Pollut. Res.* 27 45476–45486. 10.1007/s11356-020-10413-y 32794094

[B3] AbbasiK. R.ShahbazM.ZhangJ.IrfanM.AlvaradoR. (2022). Analyze the environmental sustainability factors of China: The role of fossil fuel energy and renewable energy. *Renew. Energy* 187 390–402. 10.1016/j.renene.2022.01.066

[B4] AhmadB.DaL.AsifM. H.IrfanM.AliS. (2021). Understanding the Antecedents and Consequences of Service-Sales Ambidexterity: A Motivation-Opportunity-Ability (MOA) Framework. *Sustainability* 13 9675. 10.3390/su13179675

[B5] AhmadB.IrfanM.SalemS.AsifM. H. (2022). Energy Efficiency in the Post-COVID-19 Era: Exploring the Determinants of Energy-Saving Intentions and Behaviors. *Front. Energy Res.* 9:824318. 10.3389/fenrg.2021.824318

[B6] AhukaemereC. M.OkoliN. H.AririguzoB. N.OnwudikeS. U. (2020). Tropical soil carbon stocks in relation to fallow age and soil depth. *Malaysian J. Sustain. Agric.* 4 05–09. 10.26480/mjsa.01.2020.05.09

[B7] AliS.YanQ.HussainM. S.IrfanM.AhmadM.RazzaqA. (2021). Evaluating green technology strategies for the sustainable development of solar power projects: evidence from Pakistan. *Sustainability* 13:12997. 10.3390/su132312997

[B8] BhuiyanM. A.ZamanK.ShoukryA. M.GaniS.SharkawyM. A.SasmokoS. (2018). Energy, tourism, finance, and resource depletion: panel data analysis. *Energy Sources Part B Econ. Plan. Policy* 13 463–474. 10.1080/15567249.2019.1572837

[B9] ChenQ.NingB.PanY.XiaoJ. (2021). Green finance and outward foreign direct investment: evidence from a quasi-natural experiment of green insurance in China. *Asia Pac. J. Manag.* 1–26. 10.1007/s10490-020-09750-w

[B10] ChienF.ZhangY.SadiqM.HsuC. (2021). Financing for energy efficiency solutions to mitigate opportunity cost of coal consumption: An empirical analysis of Chinese industries. *Environ. Sci. Pollut. Res. Int.* 29 2448–2465. 10.1007/s11356-021-15701-9 34374014

[B11] DebrahC.ChanA. P. C.DarkoA. (2022). Green finance gap in green buildings: A scoping review and future research needs. *Build. Environ.* 207:108443. 10.1016/J.BUILDENV.2021.108443

[B12] DmuchowskiP.DmuchowskiW.Baczewska-Da̧browskaA. H.GworekB. (2021). Green economy – growth and maintenance of the conditions of green growth at the level of polish local authorities. *J. Clean. Prod.* 301:126975. 10.1016/j.jclepro.2021.126975

[B13] DongF.ZhuJ.LiY.ChenY.GaoY.HuM. (2022). How green technology innovation affects carbon emission efficiency: evidence from developed countries proposing carbon neutrality targets. *Environ. Sci. Pollut. Res.* 1–20. 10.1007/S11356-022-18581-9/TABLES/1335061172

[B14] ElavarasanR. M.PugazhendhiR.IrfanM.Mihet-PopaL.CampanaP. E.KhanI. A. (2022a). A novel Sustainable Development Goal 7 composite index as the paradigm for energy sustainability assessment: A case study from Europe. *Appl. Energy* 307:118173. 10.1016/j.apenergy.2021.118173

[B15] ElavarasanR. M.PugazhendhiR.IrfanM.Mihet-PopaL.KhanI. A.CampanaP. E. (2022b). State-of-the-art sustainable approaches for deeper decarbonization in Europe – An endowment to climate neutral vision. *Renew. Sustain. Energy Rev.* 159:112204. 10.1016/j.rser.2022.112204

[B16] ElavarasanR. M.PugazhendhiR.ShafiullahG. M.IrfanM.Anvari-MoghaddamA. (2021). A hover view over effectual approaches on pandemic management for sustainable cities – The endowment of prospective technologies with revitalization strategies. *Sustain. Cities Soc.* 68:102789. 10.1016/j.scs.2021.102789 35004131PMC8719117

[B17] FengY.WuH. (2022). How does industrial structure transformation affect carbon emissions in China: the moderating effect of financial development. *Environ. Sci. Pollut. Res.* 29 13466–13477. 10.1007/s11356-021-16689-y 34595705

[B18] GalvãoL. S.dos SantosJ. R.RobertsD. A.BreunigF. M.ToomeyM.de MouraY. M. (2011). On intra-annual EVI variability in the dry season of tropical forest: A case study with MODIS and hyperspectral data. *Remote Sens. Environ.* 115 2350–2359. 10.1016/J.RSE.2011.04.035

[B19] GuoL.ZhaoS.SongY.TangM.LiH. (2022). Green finance, chemical fertilizer use and carbon emissions from agricultural production. *Agriculture* 12:313. 10.3390/AGRICULTURE12030313PMC922271735742399

[B20] HaoL. N.UmarM.KhanZ.AliW. (2021). Green growth and low carbon emission in G7 countries: How critical the network of environmental taxes, renewable energy and human capital is? *Sci. Total Environ.* 752:141853. 10.1016/j.scitotenv.2020.141853 32889278

[B21] HaoM.TangY.ZhuS. (2022). Effect of input servitization on carbon mitigation: evidence from China’s manufacturing industry. *Environ. Sci. Pollut. Res.* 1 1–13. 10.1007/S11356-021-18428-9/TABLES/734982390

[B22] HaoY.GaiZ.YanG.WuH.IrfanM. (2021). The spatial spillover effect and nonlinear relationship analysis between environmental decentralization, government corruption and air pollution: Evidence from China. *Sci. Total Environ.* 763:144183. 10.1016/j.scitotenv.2020.144183 33383516

[B23] HassanT.SongH.KhanY.KirikkaleliD. (2022). Energy efficiency a source of low carbon energy sources? Evidence from 16 high-income OECD economies. *Energy* 243:123063. 10.1016/J.ENERGY.2021.123063

[B24] HouD.ChanK. C.DongM.YaoQ. (2022). The impact of economic policy uncertainty on a firm’s green behavior: Evidence from China. *Res. Int. Bus. Finance* 59:101544. 10.1016/j.ribaf.2021.101544

[B25] HuJ. L.ChenY. C.YangY. P. (2022). The development and issues of energy-ICT: a review of literature with economic and managerial viewpoints. *Energies* 15:594. 10.3390/EN15020594

[B26] HuangH.ChauK. Y.IqbalW.FatimaA. (2021). Assessing the role of financing in sustainable business environment. *Environ. Sci. Pollut. Res.* 29 7889–7906. 10.1007/s11356-021-16118-0 34480700

[B27] IqbalW.TangY. M.ChauK. Y.IrfanM.MohsinM. (2021b). Nexus between air pollution and NCOV-2019 in China: application of negative binomial regression analysis. *Process Saf. Environ. Prot.* 150 557–565. 10.1016/j.psep.2021.04.039

[B28] IqbalW.TangY. M.LijunM.ChauK. Y.XuanW.FatimaA. (2021c). Energy policy paradox on environmental performance: The moderating role of renewable energy patents. *J. Environ. Manage.* 297:113230. 10.1016/J.JENVMAN.2021.113230 34303199

[B29] IqbalS.Taghizadeh-HesaryF.MohsinM.IqbalW. (2021a). Assessing the Role of the green finance index in environmental pollution reduction. *Estud. Econ. Apl.* 39. 10.25115/eea.v39i3.4140

[B30] IrfanM.AhmadM. (2021). Relating consumers’ information and willingness to buy electric vehicles: Does personality matter? *Transp. Res. Part D Transp. Environ.* 100:103049. 10.1016/j.trd.2021.103049

[B31] IrfanM.AhmadM. (2022). Modeling consumers’ information acquisition and 5G technology utilization: Is personality relevant? *Pers. Individ. Dif.* 188:111450. 10.1016/j.paid.2021.111450

[B32] IrfanM.ElavarasanR. M.AhmadM.MohsinM.DagarV.HaoY. (2022). Prioritizing and overcoming biomass energy barriers: Application of AHP and G-TOPSIS approaches. *Technol. Forecast. Soc. Change* 177:121524. 10.1016/j.techfore.2022.121524

[B33] IrfanM.ElavarasanR. M.HaoY.FengM.SailanD. (2021a). An assessment of consumers’ willingness to utilize solar energy in china: End-users’ perspective. *J. Clean. Prod.* 292:126008. 10.1016/j.jclepro.2021.126008

[B34] IrfanM.HaoY.IkramM.WuH.AkramR.RaufA. (2021b). Assessment of the public acceptance and utilization of renewable energy in Pakistan. *Sustain. Prod. Consum.* 27 312–324. 10.1016/j.spc.2020.10.031

[B35] IrfanM.RazzaqA.SuksatanW.SharifA.ElavarasanR. M.YangC. (2021c). Asymmetric impact of temperature on COVID-19 spread in India: Evidence from quantile-on-quantile regression approach. *J. Therm. Biol.* 104:103101. 10.1016/j.jtherbio.2021.103101 35180949PMC8450230

[B36] IrfanM.ZhaoZ. Y.IkramM.GilalN. G.LiH.RehmanA. (2020). Assessment of India’s energy dynamics: Prospects of solar energy. *J. Renew. Sustain. Energy* 12:053701. 10.1063/1.5140236

[B37] IslamM. M.IrfanM.ShahbazM.VoX. V. (2021). Renewable and non-renewable energy consumption in Bangladesh: The relative influencing profiles of economic factors, urbanization, physical infrastructure and institutional quality. *Renew. Energy* 184 1130–1149. 10.1016/j.renene.2021.12.020

[B38] JinY.GaoX.WangM. (2021). The financing efficiency of listed energy conservation and environmental protection firms: Evidence and implications for green finance in China. *Energy Policy* 153:112254. 10.1016/j.enpol.2021.112254

[B39] KhanH.KhanI.BiBiR. (2022). The role of innovations and renewable energy consumption in reducing environmental degradation in OECD countries: an investigation for Innovation Claudia Curve. *Environ. Sci. Pollut. Res.* 1–14. 10.1007/S11356-022-18912-W/TABLES/735119641

[B40] KhanI.HouF.IrfanM.ZakariA.PhongH. (2021). Does energy trilemma a driver of economic growth? The roles of energy use, population growth, and financial development. *Renew. Sustain. Energy Rev.* 146:111157. 10.1016/j.rser.2021.111157

[B41] KhanI.ZakariA.ZhangJ.DagarV.SinghS. (2022). A study of trilemma energy balance, clean energy transitions, and economic expansion in the midst of environmental sustainability: New insights from three trilemma leadership. *Energy* 248:123619. 10.1016/J.ENERGY.2022.123619

[B42] KhanM. A.RiazH.AhmedM.SaeedA. (2021). Does green finance really deliver what is expected? An empirical perspective. *Borsa Istanbul Rev.* 10.1016/j.bir.2021.07.006

[B43] LatifY.ShunqiG.BashirS.IqbalW.AliS.RamzanM. (2021). COVID-19 and stock exchange return variation: empirical evidences from econometric estimation. *Environ. Sci. Pollut. Res.* 28 60019–60031. 10.1007/s11356-021-14792-8 34155586PMC8216325

[B44] LeeC. C.LeeC. C. (2022). How does green finance affect green total factor productivity? Evidence from China. *Energy Econ.* 107:105863. 10.1016/J.ENECO.2022.105863

[B45] LiZ.KuoT. H.Siao-YunW.The VinhL. (2022). Role of green finance, volatility and risk in promoting the investments in Renewable Energy Resources in the post-covid-19. *Resour. Policy* 76:102563. 10.1016/j.resourpol.2022.102563

[B46] LiZ.WangJ.CheS. (2021). Synergistic effect of carbon trading scheme on carbon dioxide and atmospheric pollutants. *Sustainability* 13:5403. 10.3390/SU13105403

[B47] LiuH.TangY. M.IqbalW.RazaH. (2021). Assessing the role of energy finance, green policies, and investment towards green economic recovery. *Environ. Sci. Pollut. Res.* 1 1–14. 10.1007/S11356-021-17160-8/TABLES/9PMC857631334751878

[B48] LozanoS.GutiérrezE. (2008). Non-parametric frontier approach to modelling the relationships among population, GDP, energy consumption and CO2 emissions. *Ecol. Econ.* 66 687–699. 10.1016/J.ECOLECON.2007.11.003

[B49] MohsinM.UllahH.IqbalN.IqbalW.Taghizadeh-HesaryF. (2021). How external debt led to economic growth in South Asia: A policy perspective analysis from quantile regression. *Econ. Anal. Policy* 72 423–437. 10.1016/J.EAP.2021.09.012

[B50] MostafaM. M. (2011). Modeling Islamic banks’ efficiency: a non-parametric frontier approach. *Int. J. Islam. Middle East. Finance Manag.* 4 7–29. 10.1108/17538391111122186

[B51] NawazM. A.SeshadriU.KumarP.AqdasR.PatwaryA. K.RiazM. (2021). Nexus between green finance and climate change mitigation in N-11 and BRICS countries: empirical estimation through difference in differences (DID) approach. *Environ. Sci. Pollut. Res.* 28 6504–6519. 10.1007/s11356-020-10920-y 32997248PMC7526081

[B52] NgoT. Q. (2022). How do environmental regulations affect carbon emission and energy efficiency patterns? A provincial-level analysis of Chinese energy-intensive industries. *Environ. Sci. Pollut. Res.* 29 3446–3462. 10.1007/s11356-021-15843-w 34389945

[B53] NingY.CherianJ.SialM. S.Álvarez-OteroS.ComiteU.Zia-Ud-DinM. (2022). Green bond as a new determinant of sustainable green financing, energy efficiency investment, and economic growth: a global perspective. *Environ. Sci. Pollut. Res.* 1 1–16. 10.1007/s11356-021-18454-7 34993809PMC8735735

[B54] NuvvulaR. S. S.DevarajE.MaduraiR.ImanS.IrfanM.SrinivasaK. (2022). Multi-objective mutation-enabled adaptive local attractor quantum behaved particle swarm optimisation based optimal sizing of hybrid renewable energy system for smart cities in India. *Sustain. Energy Technol. Assess.* 49 101689. 10.1016/j.seta.2021.101689

[B55] PanD.ChenH. (2021). Border pollution reduction in China: The role of livestock environmental regulations. *China Econ. Rev.* 69:101681. 10.1016/j.chieco.2021.101681

[B56] RasoulinezhadE.Taghizadeh-HesaryF. (2022). Role of green finance in improving energy efficiency and renewable energy development. *Energy Effic.* 15 1–12. 10.1007/S12053-022-10021-4/TABLES/1135529528PMC9058054

[B57] RaufA.OzturkI.AhmadF.ShehzadK.ChandiaoA. A.IrfanM. (2021). Do tourism development, energy consumption and transportation demolish sustainable environments? evidence from Chinese Provinces. *Sustainability* 13:12361. 10.3390/su132212361

[B58] RazzaqA.AjazT.LiJ. C.IrfanM.SuksatanW. (2021). Investigating the asymmetric linkages between infrastructure development, green innovation, and consumption-based material footprint: Novel empirical estimations from highly resource-consuming economies. *Resour. Policy* 74:102302. 10.1016/j.resourpol.2021.102302

[B59] RazzaqA.SharifA.AzizN.IrfanM.JermsittiparsertK. (2020). Asymmetric link between environmental pollution and COVID-19 in the top ten affected states of US: A novel estimations from quantile-on-quantile approach. *Environ. Res.* 191:110189. 10.1016/j.envres.2020.110189 32919963PMC7483127

[B60] Saeed MeoM.KarimM. Z. A. (2021). The role of green finance in reducing CO2 emissions: An empirical analysis. *Borsa Istanbul Rev.* 22 169–178. 10.1016/j.bir.2021.03.002

[B61] ShiR.IrfanM.LiuG.YangX.SuX. (2022). Analysis of the impact of livestock structure on carbon emissions of animal husbandry: a sustainable way to improving public health and green environment. *Front. Public Heal.* 10:835210. 10.3389/fpubh.2022.835210 35223746PMC8873578

[B62] SonN. T.ChenC. F.ChenC. R.MinhV. Q.TrungN. H. (2014). A comparative analysis of multitemporal MODIS EVI and NDVI data for large-scale rice yield estimation. *Agric. For. Meteorol.* 197 52–64. 10.1016/J.AGRFORMET.2014.06.007

[B63] SrivastavaA. K.DharwalM.SharmaA. (2021). Green financial initiatives for sustainable economic growth: A literature review. *Mater. Today Proc.* 49 3615–3618. 10.1016/j.matpr.2021.08.158

[B64] SunY.SunH.MaZ.LiM.WangD. (2022). An empirical test of low-carbon and sustainable financing&rsquo;s spatial spillover effect. *Energies* 15:952. 10.3390/EN15030952

[B65] Taghizadeh-HesaryF.YoshinoN.InagakiY.MorganP. J. (2021). Analyzing the factors influencing the demand and supply of solar modules in Japan – Does financing matter. *Int. Rev. Econ. Financ.* 74 1–12. 10.1016/j.iref.2021.01.012

[B66] TangC.IrfanM.RazzaqA.DagarV. (2022). Natural resources and financial development: Role of business regulations in testing the resource-curse hypothesis in ASEAN countries. *Resour. Policy* 76:102612. 10.1016/j.resourpol.2022.102612

[B67] TanveerA.ZengS.IrfanM. (2021). Do perceived risk, perception of self-efficacy, and openness to technology matter for solar pv adoption? An application of the extended theory of planned behavior. *Energies* 14:5008. 10.3390/en14165008

[B68] TawiahV.ZakariA.AdedoyinF. F. (2021). Determinants of green growth in developed and developing countries. *Environ. Sci. Pollut. Res.* 28 39227–39242. 10.1007/S11356-021-13429-0/TABLES/11PMC831048733751350

[B69] TrubyJ.BrownR. D.DahdalA.IbrahimI. (2022). Blockchain, climate damage, and death: Policy interventions to reduce the carbon emissions, mortality, and net-zero implications of non-fungible tokens and Bitcoin. *Energy Res. Soc. Sci.* 88:102499. 10.1016/J.ERSS.2022.102499

[B70] UsmanM.JahangerA.MakhdumM. S. A.Balsalobre-LorenteD.BashirA. (2022). How do financial development, energy consumption, natural resources, and globalization affect Arctic countries’ economic growth and environmental quality? An advanced panel data simulation. *Energy* 241:122515. 10.1016/J.ENERGY.2021.122515

[B71] van VeelenB. (2021). Cash cows? Assembling low-carbon agriculture through green finance. *Geoforum* 118 130–139. 10.1016/j.geoforum.2020.12.008

[B72] WangH.LuoQ. (2022). Can a colonial legacy explain the pollution haven hypothesis? A city-level panel analysis. *Struct. Change Econ. Dyn.* 60 482–495. 10.1016/J.STRUECO.2022.01.004

[B73] WangQ.DongZ. (2022). Technological innovation and renewable energy consumption: a middle path for trading off financial risk and carbon emissions. *Environ. Sci. Pollut. Res.* 1 1–17. 10.1007/s11356-021-17915-3 35025046

[B74] WangZ.ShahidM. S.Binh AnN.ShahzadM.Abdul-SamadZ. (2022). Does green finance facilitate firms in achieving corporate social responsibility goals? *Econ. Res. Ekon. Istraživanja* 1–20. 10.1080/1331677X.2022.2027259

[B75] WenC.AkramR.IrfanM.IqbalW.DagarV.Acevedo-DuquedÁ (2022). The asymmetric nexus between air pollution and COVID-19: Evidence from a non-linear panel autoregressive distributed lag model. *Environ. Res.* 209:112848. 10.1016/j.envres.2022.112848 35101402PMC8800540

[B76] WuH.BaN.RenS.XuL.ChaiJ.IrfanM. (2021). The impact of internet development on the health of Chinese residents: Transmission mechanisms and empirical tests. *Socioecon. Plann. Sci.* 101178. 10.1016/j.seps.2021.101178

[B77] XiangH.ChauK. Y.IqbalW.IrfanM.DagarV. (2022). Determinants of social commerce usage and online impulse purchase: implications for business and digital revolution. *Front. Psychol.* 13:837042. 10.3389/fpsyg.2022.837042 35242088PMC8886314

[B78] XiongQ.SunD. (2022). Influence analysis of green finance development impact on carbon emissions: an exploratory study based on fsQCA. *Environ. Sci. Pollut. Res.* 1–12. 10.1007/S11356-021-18351-Z/TABLES/9PMC878358935066850

[B79] YanG.PengY.HaoY.IrfanM.WuH. (2021). Household head’ s educational level and household education expenditure in China: The mediating effect of social class identification. *Int. J. Educ. Dev.* 83 102400. 10.1016/j.ijedudev.2021.102400

[B80] YangC.HaoY.IrfanM. (2020). Since January 2020 Elsevier has Created a COVID-19 Resource Centre with Free Information in English and Mandarin on the Novel Coronavirus COVID- 19. The COVID-19 Resource Centre is Hosted on Elsevier Connect, The company’ s Public News and Information.

[B81] YaoX.TangX. (2021). Does financial structure affect CO2 emissions? Evidence from G20 countries. *Financ. Res. Lett.* 41:101791. 10.1016/j.frl.2020.101791

[B82] YeJ.Al-FadlyA.HuyP. Q.NgoT. Q.HungD. D. P.TienN. H. (2022). *The Nexus Among Green Financial Development and Renewable Energy: Investment in the Wake of the Covid-19 Pandemic.* 10.1080/1331677X.2022.2035241

[B83] YuM.KubiczekJ.DingK.JahanzebA.IqbalN. (2022). Revisiting SDG-7 under energy efficiency vision 2050: the role of new economic models and mass digitalization in OECD. *Energy Effic.* 15 1–20. 10.1007/S12053-021-10010-Z/TABLES/934980948PMC8716332

[B84] ZahoorZ.KhanI.HouF. (2022). Clean energy investment and financial development as determinants of environment and sustainable economic growth: evidence from China. *Environ. Sci. Pollut. Res.* 29 16006–16016. 10.1007/s11356-021-16832-9 34636020

[B85] ZengY.WangF.WuJ.ZengY.WangF.WuJ. (2022). The impact of green finance on urban haze pollution in China: a technological innovation perspective. *Energies* 15:801. 10.3390/EN15030801

[B86] ZhangD.VigneS. A. (2021). The causal effect on firm performance of China’s financing–pollution emission reduction policy: Firm-level evidence. *J. Environ. Manage.* 279:111609. 10.1016/j.jenvman.2020.111609 33218832

[B87] ZhangD.AwawdehA. E.HussainM. S.NgoQ. T.HieuV. M. (2021a). Assessing the nexus mechanism between energy efficiency and green finance. *Energy Effic.* 14 1–18. 10.1007/S12053-021-09987-4/TABLES/6

[B88] ZhangD.MohsinM.RasheedA. K.ChangY.Taghizadeh-HesaryF. (2021b). Public spending and green economic growth in BRI region: Mediating role of green finance. *Energy Policy* 153:112256. 10.1016/j.enpol.2021.112256

[B89] ZhangH.GengC.WeiJ. (2022). Coordinated development between green finance and environmental performance in China: The spatial-temporal difference and driving factors. *J. Clean. Prod.* 346 131150. 10.1016/J.JCLEPRO.2022.131150

[B90] ZhaoS.HafeezM.FaisalC. M. N. (2022). Does ICT diffusion lead to energy efficiency and environmental sustainability in emerging Asian economies? *Environ. Sci. Pollut. Res.* 29 12198–12207. 10.1007/S11356-021-16560-0/TABLES/634564809

[B91] ZhaoX.MaX.ShangY.YangZ.ShahzadU. (2022). Green economic growth and its inherent driving factors in Chinese cities: Based on the Metafrontier-global-SBM super-efficiency DEA model. *Gondwana Res.* 106 315–328. 10.1016/J.GR.2022.01.013

[B92] ZhouG.ZhuJ.LuoS. (2022). The impact of fintech innovation on green growth in China: Mediating effect of green finance. *Ecol. Econ.* 193:107308. 10.1016/J.ECOLECON.2021.107308

[B93] ZhouX.TangX.ZhangR. (2020). Impact of green finance on economic development and environmental quality: a study based on provincial panel data from China. *Environ. Sci. Pollut. Res.* 27 19915–19932. 10.1007/s11356-020-08383-2 32232752

